This article has been retracted.

# Histone methyltransferase SUV39H2 regulates LSD1-dependent CDH1 expression and promotes epithelial mesenchymal transition of osteosarcoma

**DOI:** 10.1186/s12935-020-01636-7

**Published:** 2021-01-04

**Authors:** Yingying Miao, Guifeng Liu, Lin Liu

**Affiliations:** 1 Department of Anesthesiology, Union Hospital of Jilin University, Changchun, 130033 People’s Republic of China; 2 Department of Radiology, Union Hospital of Jilin University, No. 126, Xiantai Street, Changchun, 130033 Jilin People’s Republic of China

**Keywords:** Histone methyltransferases, Suppressor of variegation 3–9 homolog 2, Lysine specific demethylase-1, E-cadherin gene, Osteosarcoma

## Abstract

**Objective:**

Osteosarcoma (OS) is a malignant tumor characterized by the direct production of bone or osteoid tissues by proliferating tumor cells. Suppressor of variegation 3–9 homolog 2 (SUV39H2) is implicated in the occurrence of OS. Therefore, we designed this study to investigate effects of SUV39H2 in OS meditated by the lysine specific demethylase-1/E-cadherin (LSD1/CDH1) axis.

**Methods:**

Clinical OS tissues and paracancerous tissues were collected for analysis of SUV39H2, LSD1 and CDH1 expression, and Kaplan–Meier survival analysis was applied to test the relationship between SUV39H2 expression and overall survival. Loss- and gain-of-function assays were conducted to determine the roles of SUV39H2, LSD1 and CDH1 in OS epithelial mesenchymal transition (EMT) and migration in OS cells, with quantitation of relevant proteins by immunofluorescence. We confirmed the effects of modulating the SUV39H2/CDH1 axis in a mouse OS tumor model.

**Results:**

SUV39H2 and LSD1 were highly expressed, while CDH1 was downregulated in OS tissues and cells. SUV39H2 expression correlated inversely with overall survival of patients with OS. SUV39H2 positively regulated LSD1 expression, while LSD1 negatively regulated CDH1 expression. SUV39H2 or LSD1 overexpression, or CDH1 silencing promoted migration and EMT, as indicated by reduced E-cadherin and dramatically upregulated Vimentin and N-cadherin of OS cells. SUV39H2 expedited the progression of OS, which was reversed by CDH1 repression in the setting of OS in vitro and in vivo.

**Conclusions:**

Collectively, our results demonstrate highly expressed SUV39H2 in OS elevates the expression of LSD1 to downregulate CDH1 expression, thereby aggravating OS, providing a potential therapeutic target for treatment of OS.

## Introduction

Osteosarcoma (OS), the primary cancer of mesenchymal tissues, is a disease of differentiation related to genetic and epigenetic factors, which prevent mesenchymal stem cells from differentiating into normal osteoblasts [1]. OS has the characteristics of high phenotypic heterogeneity, and aneuploidy, as well as a high mutation rate [2]. Prior to 1970, the treatment for OS was mainly surgical resection, but the subsequent introduction of chemotherapy remarkably improved the prognosis of patients with localized OS, such that long-term survival rates significantly increased from less than 20% to 65–70% [3]. However, the overall survival of OS patients has been stagnant for many years owing to its high resistance to chemotherapy and the high incidence of lung metastases [4]. It has been reported that promotion of epithelial mesenchymal transition (EMT) is correlated with accelerated growth of osteosarcoma OS [5], which implies that elucidating mechanism highlighting EMT may hold the key for improved treatment for OS.

Histone methylation plays an important role in affecting gene expression and genomic function, such that suppression of histone methyltransferases is a promising approach to cure multiple diseases, including cancers [6]. A prior report has highlighted the effects of histone methyltransferase in OS [7]. Suppressor of variegation 3–9 homolog 2 (SUV39H2), a member of the lysine methyltransferase SUV39 subfamily, acts by influencing the degree of H3K9 methylation, transcriptional regulation, and cell cycle [8]. SUV39H2 promotes the development of OS, given that SUV39H2 expression is significantly upregulated in OS, whereas the depletion of SUV39H2 expression by specific small interfering RNAs can dramatically suppress the growth of OS cells, leading to a significant decrease in cell survival rate [9]. Furthermore, SUV39H2 can stabilize and elevate the expression of lysine specific demethylase-1 (LSD1) by virtue of its intrinsic methylating enzyme function, such that downregulation of SUV39H2 contributes to the reduction of LSD1 protein expression [10]. LSD1 was the first histone demethylase to be identified, and is expression is often increased in a variety of tumor types [11]. Indeed, LSD1 can promote the occurrence of OS [12] and can inhibit the expression of E-cadherin (CDH1) by its demethylase function [13]. More importantly, inhibition of CDH1 promotes the migration and metastasis of OS [14]. Since the implications of the SUV39H2/LSD1/CDH1 axis in OS remain under-studied, we set about to explore the molecular mechanism of SUV39H2 in OS obtained by effects on the LSD1/CDH1 axis.

## Materials and methods

### ***Bioinformatics analysis***

We searched the expression and survival curve of histone methyltransferase SUV39H2 in The Cancer Genome Atlas (TCGA) database sarcoma samples through UALCAN (http://ualcan.path.uab.edu/) [15]. UALCAN is as a comprehensive, user-friendly, and interactive web resource for the analysis of OMICS data in malignancies. It is implemented in the PERL-CGI platform with high quality graphics of high quality using javascript and CSS. UALCAN is designed to (a) offer easy access to publicly available OMICS data in malignancies (TCGA and MET500), (b) allow users to identify biomarkers or to validate potential genes of interest using *in silico* analysis, (c) provide graphs and plots displaying gene expression and survival information of patients according to gene expression, (d) determine gene expression in molecular subtypes of breast and prostate cancer, (e) assess epigenetic mediation of gene expression through promoter methylation and relate to gene expression, (f) conduct analysis on pan-cancer gene expression, and (g) provide additional information on the genes/targets of interest by linking to HPRD, GeneCards, PubMed, TargetScan, The human protein atlas, DRUGBANK, Open Targets and the GTEx. These resources allow users to gather valuable information and data on the genes/targets of interest. OS-related genes and genes that interacted with SUV39H2 were sought using GeneCard database (https://www.genecards.org/) to predict the downstream regulators of SUV39H2. UALCAN was then applied to identify genes positively associated with SUV39H2 in OS, and the program jvenn (http://jvenn.toulouse.inra.fr/app/) was used to obtain the intersection of the above genes as candidate genes for SUV39H2 downstream regulation OS. The co-expression relationship of related regulatory genes in OS was obtained through Chipbasev2.0 website (http://rna.sysu.edu.cn/chipbase/) [16]. The minimum required interaction score was set to 0.4 to analyze the interaction relationship of OS-related genes through the bioinformatics website STRING (https://string-db.org/). In this analysis, an interaction gene corresponds to an interaction relationship. The presence of more interaction genes indicates more interaction relationships, suggesting higher core degree of the gene in question in STRING analysis results.

### ***Clinical samples***

We collected OS tissues and their corresponding paracancerous tissues of 58 patients of mean (SD) age 22.7 ± 3.6 years (range 15–30 years) who visited China-Japan Union Hospital of Jilin University from January 2011 to January 2014. None of the patients had received chemotherapy or radiotherapy before surgery. These patients were followed up for 60 months until tumor recurrence or death, and survival was analyzed using the Kaplan-Meier method. The time interval from the date of surgery to the date of death was defined as the overall survival.

### ***Cell culture and grouping***

Human OS cell lines (U2OS, HOS, MG-63) and human embryo immortalized osteoblast hFOB1.19 cells were obtained from the American Type Culture Collection (Manassas, VA, USA) [17, 18]. The frozen cells were removed and immediately placed in a thermostatic water bath held at a constant temperature of 37 °C. After the cells were thawed, they were added to a centrifuge tube supplemented with Dulbecco’s modified eagle medium (DMEM) (Procell Life Science & Technology Co., Ltd., Wuhan, Hubei, China) in the absence of newborn calf serum. After that, the cells were resuspended and centrifuged at 1500 rpm for 5 min. Then the cells on the lower layer of were added with 15% fetal bovine serum (FBS), placed in an incubator at a constant temperature of 37 °C with 5% CO_2_, and routinely passaged. The cells at the logarithmic growth were adopted in subsequent experiments.

MG-63 cells (2 × 10^5^ cells/well) were inoculated in a 6-well cell culture plate during the logarithmic growth period, and transfected when the cells were adherent to the wall and the confluence reached 30–60%, following the instructions of the Lipofectamine 2000 kit (11668-027; Invitrogen, Carlsbad, CA, USA). In brief, plasmids containing short hairpin RNA (shRNA) (sh)1-SUV39H2, sh2-SUV39H2, overexpressed (oe)-SUV39H2, oe-LSD1, sh1-LSD1, sh2-LSD1, oe-CDH1 and their negative controls (NCs) (Shanghai GenePharma Co., Ltd., Shanghai, China; add to a final concentration added of 50 nM) were diluted by addition of 250 µL of serum-free Roswell Park Memorial Institute (RPMI) 1640 medium. Then, the diluted cells were gently mixed and incubated at room temperature for 5 min. Next, 5 µL of lipofectamine 2000 was diluted by adding 250 µL of serum-free RPMI1640 medium, gently mixed and incubated at room temperature for 5 min. The two samples were mixed together and incubated at room temperature for 20 min before adding to the cell culture wells for incubation at 37 °C with 5% CO_2_ for 6 h under saturated humidity. The medium containing the transfection solution in the wells were discarded and replaced with RPMI1640 medium containing 10% FBS for subsequent experimental groupings.

### ***Reverse transcription quantitation-polymerase chain reaction (RT-qPCR)***

Total RNA was extracted from human tissues and cells according to the reagent instructions of the Trizol kit (15596-018; Invitrogen). RNA was dissolved using ultra-pure water using diethylpyrocarbonate (A100174-0005; Sangon Biotech (Shanghai) Co., Ltd., Shanghai, China). An ND-1000 ultraviolet spectrophotometer (Thermo Fisher Scientific Inc., Waltham, MA, USA) was adopted to measured RNA absorbance for calculation the RNA concentration. The RT reaction was performed following instructions in the PrimeScript RT reagent kit, and RT-qPCR was conducted by the TaqMan probe method, following kit instructions (KR011A1; Puyihua Science and Technology Co., Ltd., Beijing, China). The primer sequences are shown in Table 1. A real-time PCR instrument (Bio-Rad iQ5; Bio-Rad, Hercules, CA, USA) was used for product detection, with glyceraldehyde-3-phosphate dehydrogenase (GADPH) as the internal reference of in the analysis of SUV39H2, LSD1 and CDH1 levels using the 2^−△△CT^ calculation method, where ΔΔCT = ΔCt_experimental group_ – ΔCt_Blank group_, among which ΔCt = Ct_target gene_ – Ct_GADPH_.

**Table 1:** Primer sequences for RT-qPCR

Gene	Forward sequence (5′–3′)	Reverse sequence (5′–3′)
SUV39H2	CCCAAGCTTATGGAATATTATCTTGT	CGGGATCCGTTGAGGTAACCTCTGC
LSD1	GAAACTGGAATAGCAGAGAC	GGTGGACAAAGCACAGTATCA
CDH1	CTACGTGTCT CTATCTGCAA	AAGATCATCCT GTCCCTACTC
GAPDH	CCACTCCTCCACCTTTGAC	ACCCTGTTGCTGTAGCCA

RT-qPCR, reverse transcription quantitative polymerase chain reaction; SUV39H2, Suppressor of variegation 3–9 homolog 2; LSD1, Lysine-specific demethylase 1; CDH1, E-cadherin gene; GAPDH, reduced glyceraldehyde-phosphate dehydrogenase

### ***Western blot analysis***

Total protein in tissues or cells was extracted from radio-immunoprecipitation assay buffer containing phenylmethylsulfonyl fluoride, followed by incubation on ice for 30 min at 4 °C, and the centrifuged at 8000×*g* for 10 min to collect the supernatant. The total protein concentration was measured using a bicinchoninic acid kit. Then, 50 µg of protein was dissolved in 2× sodium dodecyl sulfonate (SDS) loading buffer and boiled for 5 min. Each of the above samples was subjected to SDS-polyacrylamide gel electrophoresis, and the proteins were transferred to a polyvinylidene fluoride (PVDF) membrane by a wet transfer method with 5% skim milk powder blocked at room temperature for 1 h. Then, the PVDF membrane was overnight incubated with diluted primary antibodies to N-cadherin (22018-1-AP, 1:1000, Proteintech, Rosemont, IL, USA), E-cadherin (ab1416; 1:50, Abcam, Cambridge, UK), Vimentin (ab8978; 1:500, Abcam), SUV39H2 (ab190870; 1:1000, Abcam), LSD1 (ab129195; 1:10,000, Abcam) and CDH1 (ab181860; 1:10,000, Abcam) at 4 °C. GADPH antibody (ab181602; 1:10,000, Abcam) was used as internal reference Then, the membrane was washed 3 times with Tris Buffered saline Tween (TBST) for 10 min each, and the membrane was incubated with horseradish peroxidase (HRP)-labeled secondary antibody of goat anti-rabbit immunoglobulin G (IgG) H & L (HRP) (ab97051; 1:2000, Abcam) for 1 h. After TBST rinsing, these antibodies were placed on a clean glass plate. The same volume of A and B liquids were taken from the enhanced chemiluminescence fluorescence detection kit (No. BB-3501, Amersham, Little Chalfont, UK), and mixed in a darkened room. The mixture was added onto the membrane and placed on a gel imager for imaging of the exposure. A Bio-Rad image analysis system was used to record images, and the membrane was analyzed with Quantity One v4.6.2 software. The relative protein content was expressed by the gray value of the corresponding protein band/the gray value of β-actin protein band.

### ***Chromatin immunoprecipitation (ChIP) assay***

The EZ-Magna ChIP A/G kit (17–371; Millipore, Billerica, MA, USA) was applied in accordance with manufacturer’s instructions. After being sonicated, the cells were centrifuged at 12,000×*g* at 4 °C for 10 min to remove the insoluble components. The cells were then added with Protein G Agarose, incubated at 4 °C for 1 h and centrifuged at 5000×*g* for 1 min to remove the supernatant. Then 10 µL of supernatant was used as “Input” and the remaining supernatant was divided into two parts, which were further treated with H3K4me3 antibody (ab185637; 1:20, Abcam) and NC rabbit anti-human IgG (ab2410; 1:25, Abcam) at 4 °C using overnight incubation. Protein G Agarose was inverted and incubated at 4 °C for 1 h to precipitate the protein-DNA complexes. Following centrifugation at 5000×*g* for 1 min, the supernatant was discarded. The non-specific complex (protein-DNA complex) was eluted, and de-crosslinked at 65 °C. The recovered and purified DNA fragments were used as amplification templates for RT-qPCR experiments, and the enrichment of H3K4me3 in the LSD1 promoter region was detected by ChIP assay [10, 12].

### ***Immunofluorescence***

Cells were grown on coverslips, fixed with 40 g/L paraformaldehyde for 15 min at room temperature, washed 3 times with phosphate buffer solution (PBS), treated with 0.2% TX-100 for 20 min, and blocked with 10% goat serum (E510009, Sangon Co., Ltd., Shanghai, China). Next, the cells were treated with antibodies to E-cadherin (ab1416; 1:50, Abcam), Vimentin (ab8978; 1:200, Abcam) and N-cadherin (22018-1-AP, 1:50, Proteintech) for overnight incubation at 4 °C. Them tetramethyl rhodamine isothiocyanate-labeled fluorescent secondary antibody of goat anti-rabbit IgG H & L (ab6718; 1:1000, Abcam) and fluorescein isothiocyanate (FITC)-labeled fluorescent secondary antibody of goat anti-mouse IgG H & L (ab6785; 1:1000, Abcam) were co-incubated for 45 min. Afterwards, the cells were mounted with Vectashield (Vector Laboratories Inc., Burlingame, CA, USA), and observed and photographed under a laser scanning confocal microscope (Olympus, Tokyo, Japan).

### ***Transwell assay***

OS cells in logarithmic growth phase were starved for 24 h. On the next day, the cells were detached, centrifuged, and resuspended with the final cell concentration of 2 × 10^5^/mL. Then, 0.2 mL of the suspension was added to the upper chamber of a Transwell, and 700 µL DMEM containing 10% pre-chilled FBS (Sangon) was added to the lower chamber. The cells were cultured in a cell incubator containing 5% CO_2_ at 37 °C. After 24 h, the Transwell chamber was removed, the cells on the upper chamber and the basement membrane where wiped away using a wet cotton swab, and the remaining cells were fixed in methanol for 30 min. Next, the cells were stained for 20 min with 0.1% crystal violet, rinsed under running water, inverted, dried naturally, and finally observed under an inverted microscope. The number of transmembrane cells was counted in five randomly selected fields of view. For the invasion assay, Matrigel was added into the upper chamber of Transwell (YB356234, Yubo Biological Technology Co., Ltd., Shanghai, China), followed by the steps as described above.

### ***Flow cytometry***

After transfection for 24 h, cells were detached with trypsin in the absence of ethylenediaminetetraacetic acid and collected in a centrifuge tube. The supernatant was discarded after centrifugation. After 3 PBS washes, the sample was centrifuged again, and the supernatant removed. Annexin-V-FITC, propidium iodide (PI) and 4-(2-hydroxyethyl)piperazine-1-ethanesulfonic acid (HEPES) were mixed at a ratio of 1:2:50 to prepare Annexin-V-FITC/PI dye liquor in accordance with the manual of the Annexin-V-FITC cell apoptosis kit (C1065, Beyotime, Shanghai, China). Portions of 100 µL dye liquor were used to suspend 1 × 10^6^ cells, followed by incubation for 15 min at room temperature. After addition of 1 mL HEPES buffer solution, fluorescence of FITC and PI were detected by activating that bandpass filters for 525 and 620 nm respectively at 480 nm wavelength for detection of cell apoptosis.

### ***MG-63 xenograft model***

A total of 32 BALB/C nude mice selected from Shanghai laboratory animal center, Chinese Academy of Sciences (aged 5–6 weeks and weighing 15–18 g) were randomly assigned into 4 groups (n = 8) and were respectively injected with MG63 cells infected with lentiviral plasmids containing oe-NC, oe-SUV39H2, oe-SUV39H2 + oe-NC or oe-SUV39H2 + oe-CDH1 (GenePharma, Shanghai, China). In brief, after MG63 cells were stably transduced with lentiviral plasmids, nude mice received subcutaneous axillary injections of 1 × 10^6^ MG63 cells. On day 8 after inoculation, we recorded the volume of the xenografted tumors. On day 24 after inoculation, the mice were sacrificed by carbon dioxide asphyxiation and the tumors were excised for subsequent analysis [19]. The tumor volume was measured once a week after inoculation, and calculated based on the following formula: (a * b^2^)/2, where a is the longest diameter and b is the shortest diameter. Finally, the volume of the transplanted tumor was recorded and the growth curve was drawn for each experimental group [20].

### ***Immunohistochemistry assay***

Paraffin sections of transplanted tumor tissues were taken for immunohistochemical analysis. In brief, the sections were deparaffinized, dehydrated with gradient ethanol, and washed with tap water for 2 min. Then the sections were treated with 3% methanol in H_2_O_2_ for 20 min and washed with distilled water for 2 min, and with 0.1 M PBS for 3 min. Following antigen retrieval, normal goat serum blocking solution (C-0005, Haoran Biological Technology Co., Ltd., Shanghai, China) was added dropwise, and the slides were placed at room temperature for 20 min, and spin-dried. Primary antibody to vascular endothelial growth factor (VEGF) (ab39256; 1:250, Abcam) was added dropwise to the slides and incubated overnight at 4 °C. The sections were washed 3 times in 0.1 M PBS for 5 min each time. Next, goat anti-rabbit IgG as secondary antibody was added and incubated at 37 °C for 20 min. The slides were next added with HRP-labeled streptavidin protein working solution (0343-10000U, Yimo Biotechnology Co., Ltd., Beijing, China), incubated at 37 °C for 20 min and visualized by addition of diaminobenzidine (ST033; Whiga Technology Co., Ltd., Guangzhou, China). After color development, the sections were washed with water, and counterstained with hematoxylin (PT001; Shanghai Bogoo Biotechnology Co., Ltd., Shanghai, China) for 1 min. Then, 1% ammonia water was adopted to restored the blue color, the slides were dehydrated with gradient alcohol, cleared with xylene, and sealed with neutral gum for microscopic examination. Five high-power microscopic fields were randomly selected from each section, and 100 cells were counted in each field. Positive cells < 10% were regarded negative, 10% ≤ positive cells < 50% were considered positive, and positive cells > 50% were intensively positive.

### ***Statistical analysis***

All data were expressed as mean ± standard deviation and analyzed by SPSS 22.0 statistical software (IBM Corp., Armonk, NY, USA) of at least three independent tests. Paired *t*-test was used for comparison of the data of carcinoma and its paracancerous tissues. The data of the other two groups were compared using unpaired *t*-test. The data comparison between multiple groups was performed using one-way analysis of variance (ANOVA), followed by Tukey’s *post hoc* test. Data of different groups at different time points were compared by repeated measures ANOVA, followed by Bonferroni *post hoc* test. The Kaplan-Meier method was used to calculate the survival rate of patients, and Log-rank test was used for difference analysis. *p* < 0.05 indicated that the difference was statistically significant.

## **Results**

### ***SUV39H2 is highly expressed in OS and is negatively correlated with overall survival***

SUV39H2 has been reported to promote the development of OS [9]. We conducted this study to explore the potential mechanism of SUV39H2 in OS. TCGA data was identified in the UALCAN database, with retrieval of expression profile and survival conditions regarding target genes in the TCGA database. We found that SUV39H2 was highly expressed in OS samples from the TCGA database through the website UALCAN (Fig. 1a). Kaplan-Meier survival analysis showed OS patients with high SUV39H2 expression had lower than did those with low SUV39H2 expression (Fig. 1b). SUV39H2 expression in OS tissues and in paracancerous tissues was examined using RT-qPCR and Western blot analysis, the results of which displayed that SUV39H2 expression in patients with OS was significantly higher than in paracancerous tissues (Fig. 1c, d). Next, SUV39H2 expression in hFOB1.19, U2OS, HOS and MG63 cells was assessed using RT-qPCR (Fig. 1e). This showed that SUV39H2 was more highly expressed in U2OS, HOS and MG63 cells than that in hFOB1.19 cells, among which MG63 cells exhibited the highest expression of SUV39H2 and were therefore selected for follow-up experiments. Then, Kaplan-Meier survival analysis was conducted to analyze the relationship between the expression of SUV39H2 and the overall survival rate of enrolled patients (Fig. 1f), which displayed lower survival rate of patients with high expression of SUV39H2 compared to patients with low SUV39H2 expression. These findings indicate that high expression of SUV39H2 may contribute to OS progression.

**Fig. 1:** The expression of SUV39H2 is upregulated in patients with OS in association with reduced survival rate. **a** SUV39H2 expression in OS and normal samples from the TCGA database detected through UALCAN website. **b** Kaplan–Meier survival curves showing the effect of SUV39H2 expression on OS patient survival from the TCGA database. **c** SUV39H2 mRNA expression in OS tissues and paracancerous tissues tested using RT-qPCR. **d** SUV39H2 protein expression normalized to GAPDH in OS tissues and paracancerous tissues tested using Western blot analysis. *p < 0.05 vs. paracancerous tissues. **e** SUV39H2 expression in hFOB1.19, U2OS, HOS and MG63 cells assessed by RT-qPCR. *p < 0.05 vs. hFOB1.19 cells. **f** The relationship between SUV39H2 expression and the overall survival rate of patients with OS (n = 58) analyzed using Kaplan-Meier survival analysis. Measurement data were expressed as mean ± standard deviation derived from at least 3 independent experiments. Paired *t*-test was used for comparison between the data of carcinoma and its paracancerous tissues. One-way ANOVA was applied for comparisons among data of hFOB1.19, U2OS, HOS and MG63 cells. Kaplan-Meier graphical analysis was used to calculate the survival rate of patients (n = 58)

### ***SUV39H2 promotes EMT and migration of OS cells***

The EMT and migration of OS cells are of great significance to the development of OS. To investigate the effect of SUV39H2 on EMT and migration of OS cells, MG63 cells were transfected with vectors expressing sh-NC, sh1-SUV39H2 and sh2-SUV39H2. RT-qPCR validated that the silencing efficiency of SUV39H2 in MG63 cells in each group met the requirements for subsequent experiments (Fig. 2a). Immunofluorescence analysis of EMT-related proteins in MG63 cells showed that silencing of SUV39H2 induced increasingly intensive E-cadherin but dramatically decreased Vimentin and N-cadherin levels (*p* < 0.05) (Fig. 2b). The results of Western blot analysis showed that the protein expression of E-cadherin in MG63 cells was significantly increased, while the expression of Vimentin, *N*-cadherin and SUV39H2 was significantly decreased upon silencing of SUV39H2 (*p* < 0.05) (Fig. 2c). Cell migration and invasion capacity was assessed by Transwell assay, which exhibited that silencing of SUV39H2 induced remarkably reduced migration and invasion ability in MG63 cells (Fig. 2d). Further flow cytometric analysis showed that silencing SUV39H2 contributed to MG63 cell apoptosis (Fig. 2e). Taken together, SUV39H2 harbors pro-migration, -invasion and -EMT action in OS.

**Fig. 2:** SUV39H2 contributes to accelerated EMT and migration of OS cells. MG63 cells were transfected with sh-NC, sh1-SUV39H2 and sh2-SUV39H2. **a** Transfection efficiency of SUV39H2 evaluated using RT-qPCR. **b** The positive rates of N-cadherin, E-cadherin and Vimentin detected using Immunofluorescence. **c** The protein expression of SUV39H2, E-cadherin and Vimentin normalized to GAPDH in MG63 cells detected by Western blot analysis. **d** Cell migration and invasion tested by the means of Transwell assay. **e** Cell apoptosis detected by flow cytometry. *p < 0.05 vs. sh-NC-transfected MG63 cells. Measurement data are expressed as mean ± standard deviation derived from at least 3 independent experiments. One-way ANOVA was conducted for comparison among multiple groups, followed by Tukey’s *post hoc* test

### SUV39H2 promotes EMT and migration of OS cells by elevating LSD1 expression

To predict the downstream regulators of SUV39H2, we identified 1,357 genes related to OS through the GeneCard database, 1,640 genes that interacted with SUV39H2, and 149 genes that were positively correlated with SUV39H2 in OS on the UALCAN website. Then, 10 candidate genes were obtained by taking the intersection of the above 3 prediction results (Fig. 3a). SUV39H2 can reportedly stabilize the expression of LSD1 by its methylase function [10], and LSD1 can promote the development of OS [12]. We found that LSD1 was highly expressed in OS samples from the TCGA database analyzed by UALCAN (Fig. 3b). A significant relationship between SUV39H2 and LSD1 expression in OS from TCGA was identified on the Chipbasev2.0 website (Fig. 3c). LSD1 expression in OS tissues and in paracancerous tissues was detected using RT-qPCR and Western blot analysis, which showed that LSD1 expression was significantly increased in OS tissues when compared with paracancerous tissues (*p* < 0.05) (Fig. 3d, e). The results of RT-qPCR revealed that LSD1 and SUV39H2 expression was notably elevated after overexpressing SUV39H2 (*p* < 0.05) (Fig. 3f). To validate the mechanism of SUV39H2 elevating LSD1 expression, we predicted that the LSD1 promoter region would be highly enriched for H3K4m3 binding through the UCSC website (http://genome.ucsc.edu/) (Fig. 3g). Transcriptional activation modified by the promoter of histone H3K4m3 may be an important reason for upregulation of LSD1 in OS. Indeed, H3K4m3 enrichment in the LSD1 promoter region was validated using the ChIP assay, which displayed that H3K4m3 enrichment was significantly boosted in oe-SUV39H2-transfected MG63 cells in comparison with that in oe-NC-transfected MG63 cells (*p* < 0.05) (Fig. 3h).

**Fig. 3:** SUV39H2 promotes the expression of LSD1, thereby accelerating EMT and migration of OS cells. MG63 cells were transfected with oe-NC, oe-SUV39H2, oe-SUV39H2 + sh-NC, oe-SUV39H2 + sh1-LSD1 or oe-SUV39H2 + sh2-LSD1. **a** Venn diagram with each circle respectively displaying the OS-related genes, genes that interacted with SUV39H2 through GeneCard and genes that were positively associated with SUV39H2 in OS by UALCAN. The middle part refers to the intersection. **b** Expression of LSD1 in OS samples of TCGA database. **c** The co-expression relationship between SUV39H2 and LSD1 in OS samples obtained using Chipbasev2.0 website. **d** LSD1 mRNA expression in OS tissues and paracancerous tissues detected using RT-qPCR. **e** LSD1 protein expression normalized to GAPDH in OS tissues and paracancerous tissues detected using Western blot analysis. *p < 0.05 vs. paracancerous tissues, n = 58. **f** The LSD1 mRNA expression in MG63 cells after overexpressing SUV39H2 detected using RT-qPCR. **g** H3K4m3 enriched in LSD1 promoter region through UCSC website. **h** H3K4m3 enrichment in LSD1 promoter region evaluated using ChIP assay. **i** The transfection efficiency of LSD1 in MG63 cells determined by RT-qPCR. **j** EMT-related protein expression in MG63 cells detected using immunofluorescence. **k** The protein expression of E-cadherin, N-cadherin, Vimentin, LSD1 and SUV39H2 normalized to GAPDH in each group detected using Western blot analysis. **l** The cell migration capacity evaluated using Transwell assay. **m** The cell apoptosis detected using flow cytometry. *p < 0.05 vs. oe-NC transfected MG63 cells and #*p* < 0.05 vs. MG63 cells co-transfected with oe-SUV39H2 + sh-NC. Measurement data were expressed as mean ± standard deviation derived from at least 3 independent experiments. Paired *t*-test was used for the data of OS tissues and paracancerous tissues, and unpaired *t*-test was used for the other two groups. The data comparison between multiple groups was performed using one-way ANOVA

To study the effect of SUV39H2 on the EMT and migration of OS cells by promoting the expression of LSD1, MG63 cells were transfected with oe-NC, oe-SUV39H2, oe-SUV39H2 + sh-NC, oe-SUV39H2 + sh1-LSD1 or oe-SUV39H2 + sh2-LSD1. The transfection efficiency of LSD1 in MG63 cells in each group was validated by RT-qPCR (Fig. 3i). EMT-related protein expression in transfected MG63 cells was detected using immunofluorescence, results of which exhibited that overexpression of SUV39H2 resulted in significantly reduced E-cadherin fluorescence intensity, but increased Vimentin and N-cadherin fluorescence intensity (*p* < 0.05), which was reversed by the co-treatment of oe-SUV39H2 and sh-LSD. The results of Western blot analysis showed that overexpressed SUV39H2 reduced E-cadherin expression but elevated that of Vimentin, N-cadherin, LSD1 and SUV39H2, all of which was abrogated by co-treatment of oe-SUV39H2 and sh-LSD (Fig. 3k). The Transwell assay revealed that cell migration capacity was significantly enhanced after SUV39H2 overexpression, which could be reversed by treatment of LSD1 knockdown and SUV39H2 overexpression (Fig. 3l). Further flow cytometric analysis showed that overexpressed SUV39H2 significantly inhibited cell apoptosis, which was restored by silencing of LSD1 (Fig. 3m). To conclude, these experimental data demonstrate that the promoting action of SUV39H2 on migration and EMT of OS cells is dependent on LSD1.

### ***LSD1 promotes EMT and migration of OS cells by downregulating the expression of CDH1***

By analyzing the interaction of OS-related genes on STRING, we found that 13 genes interacted with at least 324 genes (Fig. 4a). Next, we adopted UALCAN to inquire about the expression of these 13 genes in normal and OS samples of the TCGA database, which revealed that expression changes of EGFR, IL6, TNF, EGF and CDH1 were more significant in OS samples than in normal samples (Fig. 4b). LSD1 can inhibit the expression of CDH1 by regulating its demethylase [13]. Meanwhile, CDH1 is a widely reported gene that inhibits the migration of cancer cells and the suppression of CDH1 can promote the migration of OS to aggravate OS progression [14]. We found poor expression of CDH1 in OS samples from the TCGA database relative to that in normal samples through UALCAN (Fig. 4c). The co-expression relationship between LSD1 and CDH1 was also identified using Chipbasev2.0 (Fig. 4d). As expected, expression of CDH1 in OS tissues and paracancerous tissues from patients with OS was validated by RT-qPCR and Western blot analysis showing that CDH1 expression was significantly higher in OS tissues than in paracancerous tissues (Fig. 4e, f). Furthermore, results of RT-qPCR showed that LSD1 expression was notably upregulated after overexpressing LSD1 while CDH1 expression was significantly reduced (*p* < 0.05) (Fig. 4g). To detect the mechanism of CDH1 expression inhibition triggered by demethylase LSD1, H3K4m3 was predicted to be highly enriched in CDH1 promoter region through the UCSC website (http://genome.ucsc.edu/), suggesting that transcription of genes modified by the promoter histone H3K4m3 may be an important factor in the regulatory role of LSD1 in the downregulation of CDH1 (Fig. 4h). A ChIP assay was conducted to determinate the enrichment of H3K4m3 in CDH1 promoter region, which showed that H3K4m3 enrichment in oe-LSD1-transfected cells was significantly reduced in comparison with that in oe-NC-transfected cells (*p* < 0.05) (Fig. 4i).

**Fig. 4:** LSD1 promotes EMT and migration of OS cells by inhibiting the expression of CDH1. **a** The interactive relationship of OS-related genes analyzed using STRING. The x-axis indicates the number of interactions shared by, and the y-axis indicates the gene name. **b** Heatmap displaying genes in OS samples of TCGA database predicted using UALCAN. The x-axis represents the sample and y-axis represents the name of the gene. **c** Expression of CDH1 in OS samples of TCGA database from UALCAN. **d** The co-expression relationship between LSD1 and CDH1 identified using Chipbasev2.0. **e** Expression of CDH1 in OS tissues and paracancerous tissues from patients with OS examined using RT-qPCR. **f** Expression of CDH1 normalized to GAPDH in OS tissues and paracancerous tissues from patients with OS examined using Western blot analysis. *p < 0.05 vs.. paracancerous tissues, n = 58. **g** CDH1 expression after overexpressing LSD1 measured using RT-qPCR. **h** High enrichment of H3K4m3 in CDH1 promoter region found through the UCSC website. **i** The enrichment of H3K4m3 in CDH1 promoter region assessed using ChIP assay. **j** EMT-related protein expression tested using immunofluorescence. **k** N-cadherin, E-cadherin and Vimentin protein expression normalized to GAPDH measured using Western blot analysis. **l** Cell migration capacity detected using Transwell assay. **m** Cell apoptosis detected by flow cytometry. *p < 0.05 vs. oe-NC transfected cells. #*p* < 0.05 vs. cells co-transfected with oe-LSD1 + sh-NC. Measurement data were expressed as mean ± standard deviation derived from at least 3 independent experiments. Paired *t*-test was used for the data of OS tissues and paracancerous tissues, and unpaired *t*-test was used for the other two groups. The data comparison between multiple groups was performed using one-way ANOVA

To study the effect of LSD1 on EMT and migration of OS cells by promoting the expression of CDH1, MG63 cells were transfected with oe-NC, oe-LSD1, oe-LSD1 + oe-NC, or oe-LSD1 + oe-CDH1. EMT-related protein expression was tested using immunofluorescence, which exhibited that the fluorescence intensity of E-cadherin was significantly reduced, while that of Vimentin was significantly increased upon LSD1 overexpression (*p* < 0.05), which was reversed by CDH1 elevation (Fig. 4j). The results of Western blot analysis showed that LSD1 overexpression notably decreased CDH1 and E-cadherin expression but elevated Vimentin and LSD1 expression, which was counteracted by CDH1 elevation (Fig. 4k). Transwell assay results manifested that overexpression of LSD1 enhanced migration, but upregulation of CDH1 could override this effect brought about by LSD1 overexpression (Fig. 4l). Further flow cytometric analysis showed that overexpressed LSD1 significantly reduced cell apoptosis, which was restored by overexpression of CDH1 (Fig. 4m). To sum up, CDH1 is involved in the regulatory role of LSD1 in contribution to EMT and migration of OS cells.

### ***Overexpression of CDH1 could dampen SUV39H2-promoted tumor growth of OS***

Aiming to validate further that SUV39H2 promoted the development of OS by inhibiting CDH1 expression *in vivo*, we injected BALB/c nude mice with cells harboring lentiviral plasmids containing oe-NC, oe-SUV39H2, oe-SUV39H2 + oe-NC or oe-SUV39H2 + oe-CDH1. The tumor volume and weight of transplanted tumors increased significantly after overexpressing SUV39H2 (*p* < 0.05), whereas overexpression of CDH1 abolished these results by decreasing tumor volume and weight (*p* < 0.05) (Fig. 5a, b). SUV39H2, LSD1 and CDH1 protein expression in tumor tissues was detected using Western blot analysis (Fig. 5c), which showed that SUV39H2 and LSD1 expression was significantly enhanced, while CDH1 expression was downregulated after overexpressing SUV39H2 in mice (*p* < 0.05). Intriguingly, there was no significant changes regarding SUV39H2 and LSD1 expression (*p* > 0.05), but notable increase in CDH1 was witnessed in mice injected with cells harboring oe-SUV39H2 and oe-CDH1 (*p* < 0.05). The expression of VEGF in xenografted tumor tissues was measured using immunohistochemistry (Fig. 5d), which clarified that overexpression of SUV39H2 enhanced the expression of VEGF in xenografted tumor tissues, which was reversed by CDH1 restoration (*p* < 0.05).

**Fig. 5:** SUV39H2 facilitates the progression of OS through suppression of CDH1 expression in vivo. The BALB/c nude mice were injected with cells transduced with lentiviral plasmids containing oe-NC, oe-SUV39H2, oe-SUV39H2 + oe-NC or oe-SUV39H2 + oe-CDH1 (n = 8). **a** The representative images of transplanted tumors in nude mice. **b** Tumor volume of nude mice. **c** Tumor weight of nude mice. **d** SUV39H2, LSD1 and CDH1 expression normalized to GAPDH in tumor tissues detected using Western blot analysis. **e** The expression of VEGF in each group measured using immunohistochemistry. *p < 0.05 vs. mice injected with oe-NC-infected cells. #*p* < 0.05 vs. mice inoculated by cells transduced with oe-SUV39H2 + oe-NC. Measurement data are expressed as mean ± standard deviation derived from at least 3 independent experiments. The data comparison between multiple groups was performed using one-way ANOVA, followed with Tukey’s *post hoc* test. For data comparison among groups at different time points, repeated measures ANOVA was used

## **Discussion**

OS is one of the most prevalent primary malignant tumors of bone, mainly occurring in adolescents and in the elderly, which is characterized by high invasiveness, metastasis, and adverse outcomes [21]. The life expectancy of patients with OS has remained unchanged in the past 30 years, so there is still much to learn about the biology of this disease [2]. Accumulating studies have shown that abnormal activation of EMT can effectively drive local invasion and systemic proliferation of tumor cells [22]. Histone methyltransferases such as SETD2 are significantly implicated in OS [7]. Moreover, histone methyltransferase SUV39H2 reportedly can promote the occurrence and progression of OS [9]. Therefore, we aimed in this study to investigate the mechanism whereby SUV39H2 affects OS by meditation of the LSD1/CDH1 axis. We provide new evidence implicating that upregulation of SUV39H2 promotes the expression of LSD1 to suppress CDH1 expression, thereby stimulating the progression of OS.

Our initial experimental results indicate that SUV39H2 is highly expressed in OS and that this high expression is associated with low survival rates of patients with OS. Consistent with our research findings, the expression of SUV39H2 is significantly upregulated in OS, whereas depletion of SUV39H2 expression by specific small interfering RNA could dramatically suppress the growth of OS cells, leading to a significant decrease in cell survival rate [9]. In our subsequent experiments, we found that SUV39H2 promotes EMT and migration of OS cells. As indicated by the results, silencing of SUV39H2 decreases E-cadherin and N-cadherin but reduces Vimentin expression and restrains cell migration abilities. In line with relevant literature reports, the expression of SUV39H2 is enhanced in lung adenocarcinoma, resulting in shorter overall patient survival, suggesting that SUV39H2 has a potential role in tumorigenesis and metastasis [23]. Apart from that, the expression of SUV39H2 was significantly increased in colorectal cancer tissues, and its overexpression promotes the proliferation and metastasis of cancer cells [20]. Moreover, metastasis is the leading factor in poor outcome from OS, and EMT has been associated with carcinogenesis and shown to confer metastatic properties by enhancing cell migration, invasiveness, and resistance to apoptotic stimuli [24]. Relevant reports show that E-cadherin expression was significantly downregulated in samples from OS patient with metastasis [25]. Inhibition of E-cadherin correlated with the induction of EMT, as well as proliferation and invasion of OS cells [26]. On the other hand, N-cadherin is usually upregulated in carcinomas and is recognized as an invasion promoter [27]. Of note, N-cadherin served as downstream mechanism responsible for influence of SIRT6 exerted on growth and invasion of OS cells [28].

Moreover, our results indicate that SUV39H2 promotes EMT and metastasis of OS cells by improving the expression of histone demethylase LSD1. A prior report has addressed that SUV39H2 can stabilize and facilitate the expression of LSD1 through its intrinsic methylase function [10]. Meanwhile, LSD1 promotes the occurrence of OS and is highly expressed in several diverse mesenchymal tumors, including OS [12]. Existing research indicates that the interaction between LSD1 and other genes such as circLRP6 promotes the development of OS and advances the migratory rate of OS cells [29]. Moreover, overexpressed LSD1 downregulated the expression of E-cadherin in colon cancer, thus contributing to metastasis and poor prognosis [30]. Subsequent experiments revealed that LSD1 expedited EMT and metastasis of OS cells through suppression of CDH1 expression. LSD1 can inhibit the expression of CDH1 through its demethylase function [13]. It is worth noting that silencing of CDH1 expression enhances the proliferation and metastasis of OS cells and that NSD2 inhibits the expression of CDH1 to promote the proliferation and metastasis of OS cells [26].

## **Conclusion**

Taken above results together, SUV39H2 elevates the expression of LSD1 to restrain CDH1 expression, thereby contributing to the occurrence of OS. This study investigated the potential mechanism of SUV39H2/ LSD1/CDH1 in OS, illuminating a new molecular therapy for OS. These findings have improved our understanding on the pathogenesis of OS and provided novel potential therapeutic targets for its treatment. However, there is a need for further research to establish effective targeted molecular therapies for OS, which must eventually address the gender discrepancy in the incidence of OS [31], given that the MG-63 cells used in our study were derived from males.

## Data Availability

The datasets generated/analyzed during the current study are available.

## Abbreviations

OS: Osteosarcoma
SUV39H2: Suppressor of variegation 3–9 homolog 2
LSD1: Lysine specific demethylase-1
CDH1: Cadherin
HMTs: Histone methyltransferases
ATCC: American type culture collection
DMEM: Dulbecco’s modified eagle medium
NBCS: Newborn calf serum
FBS: Fetal bovine serum
Sh: shRNA
Oe: Overexpression
RT-qPCR: Reverse transcription quantitation-polymerase chain reaction
DEPC: Diethylpyrocarbonate
GADPH: Glyceraldehyde-3-phosphate dehydrogenase
RIPA: Radio-immunoprecipitation assay
PMSF: Phenylmethylsulfonyl fluoride
BCA: Bicinchoninic acid
SDS: Sodium dodecyl sulfonate
PBS: Phosphate buffer
TRITC: Tetramethyl rhodamine isothiocyanate
FITC: Fluorescein isothiocyanate
ANOVA: Analysis of variance
